# A Case Series of Secondary Spontaneous Pneumomediastinum and Pneumothorax in Severe COVID-19 Pneumonia

**DOI:** 10.7759/cureus.22247

**Published:** 2022-02-15

**Authors:** Peter P Staiano, Shaorinkumar Patel, Kevin R Green, Mariam Louis, Hadi Hatoum

**Affiliations:** 1 Pulmonary and Critical Care Medicine, University of Florida College of Medicine – Jacksonville, Jacksonville, USA; 2 Internal Medicine, University of Florida College of Medicine – Jacksonville, Jacksonville, USA; 3 Pulmonology, University of Florida College of Medicine – Jacksonville, Jacksonville, USA

**Keywords:** pneumothorax, high-flow nasal cannula, icu, pneumomediastinum, covid-19

## Abstract

Introduction

Pneumomediastinum and pneumothorax are uncommon complications in COVID-19 patients. The exact prevalence, etiology, and outcomes are not well known. We report a case series of patients in our institution with COVID-19 related pneumomediastinum and pneumothorax and address these questions.

Methods

We conducted a single-center retrospective chart review of patients admitted at our institution with a positive polymerase chain reaction (PCR) confirming the diagnosis of COVID-19. A cohort of 500 potential study candidates was identified, of whom eight were investigated. Demographic data, hospital course, patient co-morbidities, and outcome data were collected.

Results

Eight patients were included in our study who were identified as having an event (i.e., pneumomediastinum and/or pneumothorax) during the specified timeframe. Overall, 62% of patients were on high-flow nasal cannula with an average FiO_2_ of >70%. The average oxygen saturation//fraction of inspired oxygen (SpO_2_/FiO_2_) ratio leading up to an event was 113.7286 (range: 101.11-130.66), and all of the patients not on mechanical ventilation met the criteria for acute respiratory distress syndrome (ARDS) based on the Kigali definition with SpO_2_/FiO_2_ < 315. The three patients who developed an event while requiring mechanical ventilation both had PaO_2_/FiO_2_ < 100, consistent with severe ARDS at the time of an event. The mean time in days, counted from the day of hospital admission until an event, was 10 days (range: 3-23 days). None of the cases had documented pulmonary parenchymal disease prior to developing COVID-19. To the best of our knowledge, these events were not iatrogenic in nature.

Conclusion

Secondary spontaneous pneumomediastinum and pneumothorax are rare albeit well-documented phenomena in hospitalized patients with COVID-19 infection. Interestingly, the majority of patients in our study were on high-flow nasal cannula at the time of an event. The majority of previously published data on this topic are on those who required positive pressure ventilation; however, there have been more recent papers that also describe these events in non-mechanically ventilated patients. The exact pathophysiology remains unknown, but it is likely multifactorial, and additional studies are needed to further evaluate this phenomenon.

## Introduction

Pneumomediastinum (PM) and pneumothorax (PTX) are uncommon complications in patients with COVID-19 [1]. The exact prevalence, pathophysiology, and outcomes are not well known [1-4]. Limited data suggest that the incidence of PTX/PM ranges between 0.3% and 0.91% [1,4-5]. Furthermore, most of the patients with COVID-19 who develop these complications are on mechanical ventilation [1-6]. We described here a single-center retrospective case series reviewing COVID-19 infected patients who developed secondary spontaneous PM, PTX, or both during their hospitalization. Interestingly, the majority of these events occurred in those receiving high-flow nasal cannula (HFNC), which is not as commonly documented in the current medical literature.

## Materials and methods

We conducted a retrospective chart review of patients who were admitted to our institution with a positive polymerase chain reaction (PCR) confirming the diagnosis of COVID-19 between January 1, 2020, and November 30, 2020. We received approval for this study from our Institutional Review Board. Patients were initially identified by searching for ICD-10 (The International Classification of Diseases, Tenth Revision) diagnosis codes for “PM” and “PTX” and COVID-10 in our electronic medical record system. The inclusion criteria for the study incorporated the following requirements: age greater than 18 years old, confirmed positive for SARS-CoV-2 via PCR at the time of admission, and development of either non-traumatic PTX or PM during the hospital admission.

The PM and/or PTX events were further confirmed by searching each patient’s initial chest radiograph and/or chest computed tomography (CT) reports starting with the initial imaging report upon hospital admission. The first report that documented a PM and/or PTX event was then used. Additional data that were collected included the patient’s age, gender, race, and smoking history. In addition, co-morbidities, including history of lung disease prior to contracting COVID-19, coronary artery disease, obesity, diabetes mellitus, hypertension, atrial fibrillation, cerebrovascular accidents, and cancer were noted. Data on therapeutic interventions, ventilation modes, oxygen modalities, and outcomes were collected. Patients were followed until discharge or until they passed away.

A total of 500 patients admitted to the hospital for COVID-19 between January 1, 2020, and November 30, 2020, were identified, of whom 11 met our study criteria. Three of the patients initially identified were excluded: one was due to traumatic etiology (gunshot wound) and the other two were out of hospital transfers and the ability to review their medical records was limited. The remaining eight patients were then investigated with efforts to further characterize these phenomena and address possible etiologies as well as preventative measures to avoid these complications.

## Results

Patient characteristics are outlined in Tables 1, 2.

**Table 1:** Patient baseline characteristics CAD, coronary artery disease; HTN, hypertension; CVA, cerebral vascular accident; DM, diabetes mellitus; HLD, hyperlipidemia; HFrEF, heart failure; AAA, abdominal aortic aneurysm; Afib, atrial fibrillation; CKD, chronic kidney disease

Age (years)	Gender	Race	Co-morbidities	Smoking history	Prior lung disease
59	Male	Caucasian	None	Never smoker	No
82	Male	Caucasian	CAD, HTN, CVA, DM	Never smoker	No
54	Male	African American	None	Never smoker	No
59	Female	African American	Obesity, HTN, HLD	Former smoker	No
67	Male	Caucasian	Obesity, HTN, HLD	Former smoker	No
75	Male	African American	CAD, HFrEF, AAA, bladder cancer	Former smoker	No
67	Female	Hispanic	A.Fib, CVA, CKD, HTN	Never smoker	No
82	Female	African American	DM, HTN	Never smoker	No

**Table 2:** Description of disease progression *Days from hospital admission until event recognized on chest imaging HFNC, high-flow nasal cannula; PEEP, positive end-expiratory pressure; VT, tidal volume; RR, respiratory rate; FiO_2_, fraction oxygen; PRVC, pressure regulated volume control; PC, pressure control

Age (year)	Gender	Pneumomediastinum /pneumothorax	Days to event*	Most used oxygen modality	Oxygen modality	FiO_2_ (average)	PEEP (average)	Survival
59	Male	Pneumomediastinum	3	HFNC	90%/60L	>70	-	No
82	Male	Pneumomediastinum	14	HFNC	90%/60L	>70	-	No
54	Male	Both	13	HFNC	75%/60L	>70	-	Yes
59	Female	Pneumomediastinum	5	Ventilator	90%, PEEP 18, VT 400, RR 24	>70	18	No
67	Male	Pneumothorax	10	HFNC	90%/60L	>70	10	No
75	Male	Both	7	Ventilator	100%, PEEP 20, VT 410, RR 25 (PRVC)	>70	20	No
67	Female	Both	11	HFNC	65%/60L	50-70	-	No
82	Female	Pneumothorax	23	Ventilator	30/10/100 (PC)	>70	10	No

Figure 1 shows representative chest imaging from cases. There was a male predominance (five out of eight patients) with a mean age of 68 years old. Four patients were identified as African American, three were Caucasian, and one was Hispanic. Five patients were never smokers, and none of them were identified as having lung disease prior to contracting COVID-19 pneumonia. Two of the patients had no medical co-morbidities, and the remainder had obesity, hypertension, diabetes mellitus, atrial fibrillation, hyperlipidemia, cerebrovascular accident, and heart failure with reduced ejection fraction. One patient had an additional history of abdominal aortic aneurysm and bladder cancer. Of the eight patients included in our study who were identified as having an event (i.e., PM and/or PTX) in our cohort of 500 patients during the time frame of our study, all except one required intensive level of care at the time of initial diagnosis. The average time until an event was 10.75 days. Five patients developed either PTX or both PTX and PM. Of these five cases, four of the PTX events were unilateral and one was bilateral. Three of these cases required pigtail catheter placement to evacuate the PTX. Two of them were unilateral large right-sided PTX, and one case was of bilateral PTX with a large right-sided PTX requiring a pigtail and a trace left-sided PTX that was observed. One patient who had a large right-sided PTX required immediate intubation as a result of desaturation and increased work of breathing. None of the cases of PTX or PTX/PM developed tension PTX physiology. Six out of eight patients developed subcutaneous emphysema during their hospital course. Only one patient (who happened to develop both PM and PTX) survived hospital discharge.

**Figure 1:** Representative chest imaging from cases (A) Pneumomediastinum only. (B) Pneumothorax only. (C) Both pneumomediastinum and pneumothorax.

The majority of patients were on HFNC with an average FiO_2_ of >70%. The Kigali definition of acute respiratory distress syndrome (ARDS) was used in those who were not intubated and mechanically ventilated. The Kigali definition of ARDS is as follows: new or worsening respiratory symptoms occurring within one week of clinical insult; bilateral opacities not fully explained by effusions, lobar/lung collapse, or nodules by chest radiograph or ultrasound; and SpO_2_/FiO_2_ < 315 [7]. Based on these criteria, all of our patients who were not mechanically ventilated met the criteria for ARDS with SpO_2_/FiO_2_ well below the cutoff of 315.

The mean time in days from hospital admission until an event was 10 days (range: 3-23 days). None of the cases had documented pulmonary parenchymal disease prior to developing COVID-19. Two patients had a history of smoking.

Inflammatory markers (C-reactive peptide, erythrocyte sedimentation rate, D-dimer) were also evaluated to see if there was a significant correlation between peak levels and incidence of PM and/or PTX. However, there was no correlation, and these levels varied significantly between patients. Age, sex, history of any lung disease, and smoking history do not seem to be risk factors for the development of such events. None of our patients developed malignant PM leading to tamponade or airway compression that required video-assisted thoracoscopic surgery (VATS) or thoracotomy. All of our patients developed secondary spontaneous PM and PTX in the setting of severe COVID pneumonia. None of these events were primary spontaneous as seen in patients with a history of smoking or recreational drug use, and none were iatrogenic due to intubation, central line placement, or esophageal perforation.

## Discussion

PM refers to the presence of air in the mediastinum, which usually results from alveolar rupture due to increased intrathoracic pressure [8], whereas PTX refers to the presence of air in the pleural cavity. PM is a result of rupture along the alveolar tree, which leads to an abrupt increase in the intra-alveolar pressure. Released alveolar air centripetally dissects through the pulmonary interstitium along the bronchovascular sheaths toward the pulmonary hila, into the mediastinum, which is also known as the “Macklin effect” [9,10]. Air released during a PM event can pass through the pleura resulting in PTX [11]. Both secondary PM and PTX occur in the presence of an underlying causative etiology, which, in this case, is in the setting of COVID-19 infection.

PM and PTX remain very rare complications of severe COVID infection. Most of the reported data are on those who were receiving invasive mechanical ventilation at the time of an event; however, there is emerging data related to PM and PTX/PM in those not requiring invasive mechanical ventilation [1-4]. Since the initiation of this study, other authors have also described similar observational findings regarding the development of secondary PTX and/or PTX/PM in the setting of COVID-19 pneumonia not requiring mechanical ventilation at the time of an event. Sonia and Kumar published a case report detailing the development of PM/PTX in a 62-year-old male who was on 8L NC at the time of an event and ultimately did not require chest tube placement [12]. His only prior medical history was diabetes mellitus and hyperlipidemia, similar to our patient population. Manna et al. published a case series of 11 patients who developed subcutaneous emphysema with or without PM in those not on mechanical ventilation at the time of an event [13]. The average time until the development of an event was 13.3 days based on their data. This is comparable with our finding of an average of 10.75 days until an event.

Haberal et al. also described cases of spontaneous PM in COVID-19 who also were not receiving mechanical ventilation at the time of an event [14]. They reported seven cases out of 38,492 patients who presented to the emergency department with COVID-19. This led to a ratio of 1:5,498. The ratio at our institution based on our data was 1:100, which is a much higher occurrence than has been reported in the literature thus far. Even though the incidence is rare, it may be more common than previously thought, and in the setting of increasing oxygen requirements, progressive dyspnea or shortness of breath, or an acute change in patient condition, a high index of suspicion should be used to identify PTX and/or PM as early as possible. Intervention depends on many factors and ultimately clinician discretion regarding when to intervene when an event does occur.

Our study adds to the published data on PTX and PM events in those who were not receiving invasive positive pressure ventilation. In our study, six out of eight patients who developed PTX and/or PM were on HFNC at the time of an event. The incidence of PM/PTX in our hospital was 1.6% (8/500), which is slightly higher than previously published data of 0.3% to 0.91% [1-5]. In those who were not intubated and mechanically ventilated at the time of an event, the average SpO_2_/FiO_2_ ratio was 113.7286 (range: 101.11-130.66). The average PaO_2_/FiO_2_ ratio in those who were mechanically ventilated was 78.25, consistent with severe ARDS. All of our patients in this case series were treated with the available approved methods at that time, namely intravenous corticosteroids, remdesivir, and prophylactic anticoagulation. Self-proning was encouraged as patients could tolerate it. Those who continued to deteriorate were transferred to intensive level of care, and decision for intubation and mechanical ventilation was made based on clinical judgment. Those with persistent severe hypoxemia were offered salvage therapies on a case-by-case basis, which included proning (per PROSEVA trial protocol), either inhaled epoprostenol or inhaled nitric oxide, and extracorporeal membrane oxygenation (ECMO) team consultation for veno-venous ECMO.

Furthermore, all of our patients who developed clinically significant PTX (three out of five cases of PTX or PTX/PM) were treated with pigtail catheter insertion along with supportive care, including intubation for respiratory failure (one case) and decreasing positive end-expiratory pressure (PEEP) as low as possible in mechanically ventilated patients. Similar to already published data, 75% of our patients developed subcutaneous emphysema, which, in those with PM, occurs in 70% of PM cases [9]. In those with clinically significant subcutaneous emphysema, superficial incisions or subcutaneous peripheral IVs were placed to decompress air. In addition, the mortality rate observed in our institution was 87.5%, which is consistent with previously published data that have ranged between 49% and 87.5% [2-6].

The exact pathogenesis for secondary spontaneous PM and PTX in the setting of COVID ARDS remains unknown. In particular, the occurrence of these events in patients who are not mechanically ventilated is intriguing. Based on the published data with regard to the development of PM or PTX/PM, the etiology remains elusive. However, the underlying pathophysiology is most likely multifactorial. First, increased alveolar pressure due to alveolar occlusion and destruction from diffuse alveolar damage (DAD) and ischemic microangiopathy of the lung parenchyma caused by severe inflammation could lead to bleb formation and rupture. This results in air dissecting through mediastinal fascial planes [10] In addition, increased airway pressure from coughing can exacerbate the above problem and induce the formation of PM and PTX [10]. Indeed, a review of the autopsy data published thus far confirmed the increased prevalence of DAD in patients who died due to COVID-19 [15]. Other findings from this study included microthrombi within pulmonary capillaries (despite being on anticoagulation), superimposed bacterial pneumonia, pneumocyte desquamation, and destruction of hyaline membranes, among others [15]. However, no autopsy data specifically reported findings unique to PM and PTX.

Another possible mechanism includes patient self-inflicted lung injury (P-SILI). The mechanism of P-SILI is highly debated and has more recently been brought into the spotlight due to the respiratory complications seen in COVID-19, such as PM/PTX. Strong inspiratory efforts and an increased transpulmonary pressure gradient may lead to worsening lung damage that could contribute to the formation or progression DAD [16]. Weaver et al. used computational simulations to evaluate the potential for self-induced lung injury based on multiple respiratory variables and pathophysiologic conditions [16]. They observed large changes in transpulmonary pressure, pleural pressure, and lung strain that were on par with ventilator-induced lung injuries. Their study was limited to solely spontaneous breathing with supplemental oxygen, and non-invasive ventilation effects were not investigated. However, based on these findings, it is feasible for patients to generate such a large respiratory effort as to self-induce lung injury that can lead to spontaneous PM and PTX. Battaglini et al. recently wrote a review article highlighting four potential mechanisms for P-SILI, some of which were previously mentioned [17]. These include increased lung strain/stress, heterogeneous distribution of ventilation, changes in lung perfusion, and ventilator asynchronies during non-invasive positive pressure ventilation. The complexity of COVID-19 respiratory failure has provided an opportunity to further appreciate the clinical significance of P-SILI.

The third possible mechanism by which PM/PTX complicates COVID-19 infections includes mediastinitis (viral or superimposed bacterial mediastinitis). This, in turn, may lead to the formation of PM and subsequently PTX. However, this is typically observed in cavitary pneumonia due to gas-forming organisms [18]. Currently, no published autopsy data detail the occurrence of mediastinitis in the setting of COVID-19 pneumonia.

Although to date there are no proven measures to decrease the development of PTX/PM in COVID-19 infections, several plausible considerations may be implemented based on existing literature. Measures to mitigate P-SILI should be implemented as tolerated. These measures include (1) limiting the tidal volume and respiratory effort (although difficult to achieve in clinical practice, especially those not receiving mechanical ventilation), (2) safe PEEP levels titrated to individual effect and adequate gas exchange, and (3) early recognition of those requiring intubation and mechanical ventilation to alleviate extreme work of breathing [17]. Titrating non-invasive ventilation settings to promote safer practice should be pursued as tolerated; however, as previously stated, there is potential for self-induced lung injury in those spontaneously breathing not on non-invasive modes of ventilation. Anecdotally, however, these measures seem to provide little benefit in terms of preventing the development of PM/PTX. In addition, it was previously thought that avoidance of excessive oxygen and exposure to supraphysiological PaO_2_ should be applied in an effort to not exceed normoxia and avoid the potential for oxygen toxicity. However, studies in the critically ill population do not coincide with this. Indeed, in 2020, both the ICU-ROX and LOCO2 investigators published studies evaluating conservative oxygen use in the ICU population (these patients received mechanical ventilation) [19,20]. Both studies showed neither a mortality benefit nor a reduction in ventilator-free days with the use of a conservative oxygen strategy [19,20]. Therefore, aggressively titrating FiO_2_ to adhere to conservative oxygenation may not be as clinically relevant as previously thought.

Our study has several limitations. First, it was a retrospective chart review during a specific time period during the COVID-19 pandemic. It is not clear how different COVID variants may have different clinical pulmonary manifestations. Second, our study was conducted in a single center, which may not be fully applicable to other institutions. Finally, our findings may differ if we included the entire caseload at our institution since the pandemic began, as patient demographics have changed with evolving surges.

## Conclusions

In conclusion, secondary spontaneous PM and PTX are rare albeit well-documented phenomena in hospitalized patients with COVID-19 infection, especially those requiring the intensive level of care. Conclusions cannot be drawn from our data alone, but we hope to contribute to the ongoing research regarding this specific complication from COVID-19 pneumonia. Our study adds to the emerging literature on those who have PTX/PM while not on invasive positive pressure ventilation. The exact pathophysiology remains unknown but is likely multifactorial, and further studies are needed to determine best practice strategies to prevent the development of these complications.
